RETRACTED

# Trapping mosquitoes using milk products as odour baits in western Kenya

**DOI:** 10.1186/1756-3305-3-55

**Published:** 2010-06-24

**Authors:** Eunice A Owino

**Affiliations:** 1 School of Biological Sciences, University of Nairobi, P.O. Box 30197 - 00100, Nairobi, Kenya; 2 International Center for Insect Physiology and Ecology, P.O. Box 30772 - 00100, Nairobi, Kenya

## Abstract

**Background:**

Ample evidence has shown that blood seeking mosquitoes locate their hosts by following odours produced by the hosts. Odour baited traps would therefore, provide a solution in controlling diseases spread by mosquitoes. Comparative studies were undertaken to determine the relative efficacies of two odour baits i.e. Limburger cheese and African traditional milk cream in trapping mosquitoes in the field in western Kenya.

**Method:**

Comparative efficacy studies were carried out in the field using Latin square experimental designs. In the first study, a counterflow geometry (CFG) trap (MM-x model; American Biophysics Corp., USA.) baited with Limburger cheese, man landing catches (MLC), Centres for Disease Control (CDC) light trap and an entry trap were compared. In the second study, three CFG traps baited with either Limburger cheese, African traditional milk cream or with no bait were compared and in the third study four CDC traps baited with either Limburger cheese, African traditional milk cream, light or with no bait were compared. Parameters like species, catch size, abdominal status, parity status and size of the collected mosquitoes were compared.

**Results:**

A total of 1,806 mosquitoes were collected (60% *An. gambiae s.l *and 25% *An.funestus*, culicines 15%). There was no significant difference in the number of *An. funestus *trapped by the CFG trap baited with Limburger cheese from those trapped by the MLC (P = 0.351). The Limburger cheese baited CFG trap collected significantly more gravid *An. funestus *than the MLC (P = 0.022). Furthermore, when the CFG trap baited with Limburger cheese and the CFG trap baited with milk cream were compared, there was no significant difference in the number of *An. funestus *collected (P = 0.573). The same trend was observed in the comparison of Limburger cheese baited CDC trap and milk cream baited CDC trap.

**Conclusions:**

Limburger cheese and African traditional milk cream have a potential as effective odour baits for sampling/surveillance and as oviposition attractants for the malaria vector, *Anopheles funestus*.

## Background

Ample evidence has shown that host-seeking female mosquitoes mainly locate their hosts by odours produced by the hosts [1-5]. It could, therefore, be useful if traps baited with host odours would lure mosquitoes as strongly as normal healthy humans [5] or even lure more mosquitoes than healthy human beings [6]. Such traps could then be used in the trapping of mosquitoes in large numbers [7]. This would lead to the control of infection and transmission rates of diseases spread by mosquitoes like malaria, rift valley fever and bancroftian filariasis.

RETRACTED

Current efforts centre on searching for new attractants and attractant formulations [6-8] improving on existing ones [9-11], and developing trapping devices [7,12,13]. Efficacy trials under field [14] and semi-field conditions are also on-going [15].

The demonstration that Limburger cheese, which to the human nose has a smell reminiscent of foot odour, was a strong attractant to *Anopheles gambiae *Giles *sensu stricto *[16] and to *Aedes aegypti *[17] in wind tunnel bioassays, together with the successful development and use of synthetic host odour blends in semi-field [8,14] and field conditions [6,15,17] have shown that traps based on synthetic[6-8] host attractants are likely to provide an objective monitoring tool for the host-seeking fraction of mosquito vectors of diseases like malaria and bancroftian filariasis. Such traps can be used to study the vector biology and epidemiology of mosquito-borne diseases, knowledge of which is vital for planning and assessing outcome of intervention strategies. One might even foresee the development of synthetic odour baited mosquito traps [6,7] that might be used to reduce the vector population in a village or in an individual's bedroom to divert mosquitoes away from occupants. Such traps could eventually become part of primary healthcare systems. Therefore, in an effort to look for an effective synthetic odour bait that can be used in sampling and control of disease spreading mosquitoes, comparative efficacy studies using CFG traps and CDC traps baited with either Limburger cheese or African traditional milk cream were conducted in western Kenya.

## Methods

### Ethics statement

A written institutional ethical clearance to do this study was obtained from the joint University of Nairobi/Kenyatta National Hospital Ethics and Research Committee. Verbal consents from household heads of the houses used in this study were received only after informing them of the rationale and methodology of the research work. Moreover, thick and thin blood smears were taken from the person performing the man-landing catches whenever he complained of fever to examine the presence of malaria parasites. When found positive, he was treated with Coartem^® ^(artemether-lumefantrine).

### Study Area

#### Study sites

The current study was carried out at Lwanda Nyamasari village, located along the southern shores of Lake Victoria in Suba District, western Kenya. Suba district lies at an altitude of 1100 - 1300 metres above sea level and experiences high temperatures (17 - 34°C) throughout the year. The district also experiences two rainy seasons: the long rains occur from March to June, and the short rains from September to November. The annual rainfall ranges between 700 - 1200 mm [18]. Malaria is holoendemic in Suba district and is the leading cause of morbidity, childhood mortality and hospital admissions. Transmission of the disease is maintained by three main vectors: *An. gambiae, An. arabiensis *and *An. funestus *which breed in natural and artificial larval habitats [18,19]. Malaria transmission fluctuates throughout the year and reaches its climax in the rainy seasons.

RETRACTED

#### Preliminary investigations

The efficacy of a counter flow geometry (CFG) trap baited with Limburger cheese, an entry trap, a Centers for Disease Control (CDC) light trap and man-landing catches (MLC) performed by a twenty four year-old male in sampling African malaria vectors was evaluated by comparing the species diversity, the number of mosquitoes collected, the abdominal status, the parity status and the sizes of mosquitoes collected by each method. These investigations were carried out during the dry month of January up to mid February because it was important for the CFG traps baited with Limburger cheese to be able to sample mosquitoes in low densities.

A 4 × 4 Latin square experimental design was formulated, whereby four houses were selected after obtaining a verbal consent from the heads of households. All occupants of the experimental houses were provided with untreated mosquito bed nets and asked to sleep under them. All experiments began at 22.00 and concluded at 06.00 hours on each experimental night. The CDC and the CFG traps were suspended 20 cm above the ground. In the case of the Limburger cheese baited CFG trap, 0.6 g of Limburger cheese was wrapped in a small piece of mosquito netting material and suspended inside the thin inner PVC pipe of the CFG trap so that the cheese odour could be pumped to the exterior when the fan in the trap was operated. An entry trap, measuring 0.3 × 0.3 × 0.3 m with a circular aperture of 5 cm in diameter at its center, was fixed on an open window in the sitting room of the experimental house. In the case of the man- landing technique, a 24 year-old man, who acted as both bait and collector, sat upright in the sitting room and exposed his legs. He collected every mosquito that landed on him, albeit before they could bite him.

Trapped mosquitoes were transported to the ICIPE-Mbita laboratories for processing where mosquitoes were killed using chloroform and all non-target insects discarded.

RETRACTED

Mosquitoes were identified morphologically into anophelines according to the protocol of Gillies and De Meillon [20] and Gillies and Coetzee [21] and into culicines according to the protocol of Service [22]. The abdominal status of each individual trapped mosquito was assessed into three classes "fed", "unfed" and "gravid (heavy with eggs)" according to the World Health Organization manual [23]. In preliminary studies, *Anopheles gambiae *complex mosquitoes were identified into species by the Polymerase Chain Reaction (PCR) method according to the protocol of Scott *et al. *[24]. The mosquito size was determined by pulling off the left wing of each mosquito, mounting it on a glass slide and measuring the wing length from the distal end of the alula to the tip excluding the fringe scales using an ocular micrometer that had been mounted on the eye piece of a light microscope at the magnification of × 40. The reading, which was in micrometers (μm) was then multiplied by 0.025 which was the conversion factor for the micrometer. The product was then taken as the size of the mosquito. Determination of mosquito parity status into parous (mosquitoes that have ever laid eggs) and nulliparous (mosquitoes that have never laid eggs) was performed according to the method of Detinova [25] whereby a small cut was made on the 6^th ^and the 7^th ^segment of the mosquitoes' abdomen to remove the ovaries. The tracheoles of the ovaries were examined under the low power x40 of a compound microscope. When the tracheoles were dilated at the distal end, the mosquito was termed as parous, while when the tracheoles were coiled and not dilated at the distal end; the mosquito was termed as nulliparous.

### Comparative efficacy of Limburger cheese and Milk cream as odour baits for sampling mosquitoes

#### Making Milk cream

Milk cream was made by adding 20 ml of fermented cow urine into a gourd that had been cleaned using water and soap and left in the sun until dry. Milk was then poured into the gourd and left therein for twelve hours. The gourd with the milk was churned until some cream formed on the surface of the milk. This cream is what is referred to as milk cream in this paper. The milk cream was separated from the milk and stored at 24°C in a plastic container filled with water.

##### Comparative efficacy using CFG traps

The efficacy of a milk cream baited CFG trap, a Limburger cheese baited CFG trap and an unbaited CFG trap was compared by studying the species diversity, the catch size and the abdominal status of trapped mosquitoes. A 3 × 3 Latin square design was formulated whereby three of the houses used in the preliminary investigations were used such that each method of trapping was tested separately in each one of the three houses per night until each method had been applied three times per house. The CFG traps were either baited with milk cream, Limburger cheese or unbaited. When baited, 0.6 g of Limburger cheese or milk cream was wrapped in a small piece of mosquito netting material and suspended inside the thin inner PVC pipe of the Counterflow Geometry (CFG) trap so that odours of the cheese or milk cream could be pumped to the exterior when the fan in each CFG apparatus was operated. All the CFG traps were suspended 20 cm above ground level.

RETRACTED

##### Comparative efficacy using CDC light traps

In the third series of comparative studies, the relative efficacies of a CDC light trap with light on, a CDC light trap with no light, a CDC light trap with no light but baited with Limburger cheese and a CDC light trap with no light but baited with milk cream were compared using a 4 × 4 Latin square experimental design. The four houses used in preliminary investigations were used and each sampling method was rotated four times per house.

In the cases of the CDC light trap baited with Limburger and the CDC light trap baited with milk cream, the light bulbs in each trap were removed and replaced with 0.6 g of Limburger cheese or milk cream. The CDC light traps were then suspended 20 cm above the ground.

All experiments began at 22.00 and concluded at 06.00 hours on each experimental night. All occupants of the experimental houses were provided with untreated mosquito bed nets and asked to sleep under them. Trapped mosquitoes were transported to the ICIPE-Mbita laboratories for processing as explained under the preliminary investigations. However, PCR on anopheline mosquitoes, parity status and mosquito size were not determined for these mosquitoes.

### Statistical analysis

Data were analyzed using PASW Statistic 17 (SPSS version 17). The mean mosquito catch per trap per night were first calculated and compared using either bar graphs showing 95% confidence intervals or tables. Further analysis was conducted using General Linear Model (GLM), univariate analysis of variance procedure as follows: mosquito catches were modeled as a function of trapping method as the fixed factor in both the case where the distribution of each mosquito species per trap was analyzed and also in the case where the distribution per trap of each of the three abdominal status (fed, gravid, unfed) for each mosquito species was compared. Each time 'day' was treated as a random variable to reflect daily fluctuations in mosquito numbers. To maintain validity of assumptions for appropriate data analysis, the mosquito catch were log_10 _(x +1) transformed to normalize prior to statistical analysis. For mosquito wing length comparisons, the wing length was modeled as a function of trap as the fixed factor.

RETRACTED

## Results

### Preliminary investigations

#### Analysis by mosquito species and sample size

The mean catches for each mosquito species trapped by each method per night are shown in Figure 1. It was observed that the trapping method had significance in the trapping efficacy for the mosquito species *An. arabiensis *(F = 16.713, df 3, P < 0.001), *An gambaie *(F = 13.224, df 3, P < 0.001) and *An. funestus*, (F = 11.522, df 3, P < 0.001). There was no significant difference between the *An. arabiensis *collected by the CDC light trap and the MLC, (P = 0.113). This same trend was seen for the *An. gambiae *and *An. funestus *mosquitoes. However, the CDC light trap and the MLC collected significantly more *An. arabiensis *than the CFG trap baited with Limburger cheese, (P < 0.001, 0.002) respectively and the Entry trap, (P < 0.001, 0.001) respectively. This same trend was seen for *An. gambiae *mosquitoes only that the CFG trap baited with Limburger cheese also collected significantly more *An. gambiae *than the entry trap (P = 0.042). There was no significant difference in the number of *An. funestus *collected by the CFG trap baited with Limburger cheese from those collected by the MLC (P = 0.351) while the CDC light trap collected significantly more *An. funestus *than the CFG trap baited with Limburger cheese (P = 0.043). The entry trap did not catch any *An. funestus *mosquitoes.

**Figure 1:** **Comparison of different trapping methods used in the preliminary investigations**. Average number of female anophelines caught per trap per night. The alphabetical symbols, **a, b and c **are used to represent differences as determined by unianova test. Trapping efficiencies for the different trapping methods in collecting a certain species are not significantly different (P = 0.05), if the bars representing a particular species in each trap share any of these alphabets. The Y-error bars represent 95% confidence intervals. **CFG**, Counterflow geometry trap baited with Limburger cheese; **CDC**, standard centers for disease control light trap; **ET**, Entry trap; **MLC**, man landing catches.

Day had no significance in the trapping efficacy for *An. arabiensis *(F = 1.769, df 15, P = 0.071), *An. gambiae *(F = 1.619, df 15, P = -0.107) and *An. funestus *(F = 1.454, df 15, P = 0.165).

The mean catches per trap per night for every abdominal status for the different mosquito species are shown in Table 1. The trapping method had significance in the trapping efficacy for fed *An. arabiensis *(F = 3.575, df 3, P = 0.019) and fed *An. funestus *(F = 3.000, df 3, P = 0.037) but not for fed *An. gambiae *(F = 2.277, df 3, P = 0.089). The MLC had significantly more fed *An. arabiensis *than the CDC light trap (P = 0.002), the CFG trap baited with Limburger cheese, (P = 0.002) and the entry trap (P = 0.002). This same trend was followed for *An. funestus *mosquitoes while the CFG trap baited with Limburger cheese and the entry trap did not collect any fed *An.gambiae *mosquitoes.

RETRACTED

**Table 1:** Comparison of the mean catch per trap per night for each of the three abdominal status of every mosquito species collected by the four trapping methods used in the preliminary investigations at Lwanda Nyamasari village.

		*Anopheles arabiensis*				*Anopheles gambiae*				*Anopheles funestus*				Total No. of mosquitoes %
			
Method	N	Fed mean	Unfed mean	Gravid mean	Sum %	Fed mean	Unfed mean	Gravid mean	Sum %	Fed mean	Unfed mean	Gravid mean	sum %	
CFG	16	0.2^b^	0.4^c^	0.0^a^	10 (9)	0.0^a^	1.0^b^	0.1^a ^	16 (15)	0.0^b^	2.3^a^	0.4^b^	44 (23)	70 (17)

CDC	16	0.2^b^	3.4^a^	0.1^a^	59 (51)	0.3^a^	2.1^a^	0.1^a^	40 (36)	0.0^b^	5.3^c^	0.2^ab^	89 (47)	188 (45)

ET	16	0.1^b^	0.1^c^	0.0^a^	3 (3)	0.0^a^	0.1^b^	0.0^a^	2 (2)	0.0^b^	0.0^b^	0.0^a^	0 (0.0)	5 (1)

MLC	16	0.7^a^	2.0^b^	0.1^a^	43 (37)	0.4^a ^	2.8^a^	0.1^a^	52 (47)	0.3^a^	3.2^ac^	0.1^a^	57 (30)	152 (37)

Sum of each mosquito species in each trap is also shown with the percentage in parenthesis. **CFG**, counterflow geometry trap baited with Limburger cheese; **CDC**, standard centers for disease control light trap; **ET**, entry trap; **MLC**, man landing catches; **N **represents the number of days over which sampling was done. The percentages are calculated for each mosquito species. For example the CFG trap collected 9% of all the *An. arabiensis *collected by the four trapping methods while the CDC light trap collected 51% of the same. Values following each other in the same column with different letter superscripts are significantly different at (P = 0.05).

The trapping method had significance in the trapping efficacy for gravid *An. funestus *(F = 3.078, df 3, P = 0.034) mosquitoes whereby the CFG trap baited with Limburger cheese collected significantly more gravid *An. funestus *than the (MLC P = 0.022). However, the trapping method had no significance in the trapping efficacy for gravid, *An. arabiensis *(F = 1.279, df 3, P = 0.290) and gravid *An. gambiae*, (F = 0.699, df 3, P = 0.565).

The trapping method had significance in the trapping efficacy for the unfed *An. arabiensis *(F = 15.614, df 3, P < 0.001), unfed *An. funestus *(F = 10.365, df 3, P < 0.001) and unfed *An. gambiae *(F = 10.374, df 3, P < 0.001). The CDC light trap collected significantly more unfed *An. arabiensis *than the CFG trap baited with Limburger cheese, (P < 0.001), the MLC (P = 0.019) and the entry trap, (P < 0.001). The MLC also collected significantly more unfed *An.arabiensis *than the CFG trap baited with Limburger cheese and the entry trap.

RETRACTED

The CDC, the CFG trap baited with Limburger cheese and the MLC collected significantly higher numbers of unfed *An. gambiae *than the Entry trap (P < 0.001, P = 0.021 and P < 0.001) respectively. Furthermore, the MLC collected significantly more unfed *An. gambiae *mosquitoes than the CFG trap baited with Limburger cheese (P = 0.007). However, there was no significant difference in the number of unfed *An. gambiae *collected by the CDC trap and the CFG trap baited with Limburger cheese (P = 0.541)

The CDC light trap collected higher numbers of unfed *An. funestus *than the CFG trap baited with Limburger cheese, (P = 0.021) while there was no significant difference between the unfed *An. funestus *collected by the MLC and the CFG trap baited with Limburger cheese, (P = 0.255).

#### Analysis by mosquito parity status

A total of 313 female anopheline mosquitoes were dissected in order to determine their parity status. In general, the total proportion of parous anophelines caught by the CDC light trap, CFG trap baited with Limburger cheese and man-landing catches was proportionally higher than the nulliparous anophelines collected (Table 2). The CFG trap collected higher proportions of parous *An. arabiensis*, *An. gambiae *and *An. funestus *than the CDC light trap, the entry trap and the man landing catches.

**Table 2:** Comparison of parity rates of dissected mosquitoes for the four trapping methods used in the investigations at Lwanda Nyamasari village.

	*Anopheles arabiensis*				*Anopheles gambiae*				*Anopheles funestus*			
**Method**	**Parous** **%**	**Nulli** **Parous**, **%**	**Not dissected, %**	**Sum**	**Parous, %**	**Nulli** **Parous,%**	**Not** **dissected, %**	**Sum**	**Parous,%**	**Nulli** **Parous, %**	**Not dissected %**	**sum**

CFG	80%	0%	20%	10	69%	19%	12%	16	66%	30%	4%	44

CDC	66%	15%	19%	59	63%	15%	22%	40	48%	15%	37%	89

ET	0%	67%	33%	3	50%	0%	50%	2	0%	0%	0%	0

MLC	49%	19%	33%	43	60%	17%	23%	52	55%	18%	27%	57

**CFG**, counterflow geometry trap baited with Limburger cheese; **CDC**, standard centers for disease control light trap; **ET**, entry trap; **MLC**, man landing catches; The percentages are calculated for each mosquitoes species per trap. For example, of all the *An. arabiensis *mosquitoes collected by the CFG trap, 80% were parous while of all the *An. arabiensis *mosquitoes collected by the CDC light trap 66% were parous.

RETRACTED

#### Analysis by mosquito size

Size was determined for all the mosquitoes collected. Trap had a significant influence on the wingsize of *An. arabiensis *(F = 9.328, df 3, P < 0.001) and *An. gambiae *(F = 5.231, df 3, P = 0.002) but not for *An. funestus *(F = 0.413, df 2, P = 0.662) collected by the different trapping methods.

The man-landing catches collected bigger *An. arabiensis *than the CDC light trap (P < 0.001) and the CFG trap baited with Limburger cheese (P = 0.001) while the CDC light trap had smaller *An. gambiae *than the CFG trap baited with Limburger cheese, (P = 0.001) and the MLC, (P = 0.002) (Table 3).

**Table 3:** Comparison of mean wingsize (Measurements in micrometers) for each anopheline species collected by the four sampling methods used in the preliminary investigations at Lwanda Nyamasari village.

	*Anopheles arabiensis*		*Anopheles funestus*		***Anopheles gambiae***.	
**Trap**	**Mean Wingsize/trap**	**± SD**	**Mean Wingsize/trap**	**± SD**	**Mean Wingsize/trap**	**± SD**

CDC	2.0(59)^b^	0.34	2.1(89)^a^	0.28	2.0(40)^a^	0.26
CFG	2.0(10)^b^	0.23	2.1(44)^a^	0.51	2.4(16)^b^	0.46
ENTRY	2.3(3)^ab^	0.46	0	0	2.1(2)^ab^	0.85
MLC	2.4(43)^a^	0.36	2.0(57)^a^	0.35	2.3(52)^b^	0.36

Sum of mosquitoes is in parenthesis.

**CDC**, standard centers for disease control light trap; **CFG**, counterflow geometry trap baited with Limburger cheese; **ET**, entry trap; **MLC**, man landing catches.

Values following each other in the same column with different letter superscripts are significantly different at (P = 0.05).

#### Comparative efficacy studies using CFG traps

The mean catches of mosquitoes for each species trapped by each trapping method per night are shown in Figure 2. The trapping method had significance on the trap efficacy in trapping *An. funestus *(F = 3.022, df 2, P = 0.055) and the culicine mosquitoes (F = 3.473, df 2, P = 0.036) but it had no significance on trap efficacy in trapping *An. gambiae*, (F = 2.574, df 2, P = 0.083). There was no significant difference in the number of *An.funestus *collected by the CFG trap baited with Limburger cheese and the CFG trap baited with milk cream (P = 0.573). This trend was followed for the *An. gambiae s.l *mosquitoes and the culicine mosquitoes. However, the Limburger cheese baited trap collected significantly higher numbers of *An. funestus *than the trap with no bait, (P = 0.021) while there was no significant difference in the number of *An*. *funestus *collected by the milk cream baited trap, (P = 0.078) and the trap with no bait. Also, the milk cream baited trap had significantly more *An. gambiae *than the trap with no bait (P = 0.031) while there was no difference in the number of *An. gambiae *collected by the Limburger cheese baited trap and the no bait trap (P = 0.122). The trap with no bait collected significantly lower numbers of culicines than the trap baited with milk cream P = 0.036 and the trap baited with Limburger cheese P = 0.019

**Figure 2:** **Comparison of different trapping methods used in the comparative studies by counterflow geometry traps**. Average number of female mosquitoes caught per trap per night. The alphabetical symbols, **a**, **b **are used to represent differences as determined by unianova test. Trapping efficiencies for the different trapping methods in collecting a certain species are not significantly different (P = 0.05), if the bars representing a particular species in each trap share any of these alphabets. The Y-error bars represent 95% confidence intervals. **CFG LC**, counterflow geometry trap baited with Limburger cheese; **CFG MC**, counterflow geometry trap baited with milk cream; **CFG NB **counterflow geometry trap NOT baited.

RETRACTED

Day had no significance in the trapping efficacy for *An. funestus *(F = 0.412, df 8, P = 0.910), *An. gambiae*, (F = 0.608, df 8, P = 0.768) and culicines (F = 0.265, df 8, P = 0.975).

The mean catches per trap per night for every abdominal status for the different mosquito species are shown in Table 4. The trapping method had no significance on the trap efficacy in trapping fed *An. funestus *(F = 1.091, df 2, P = 0.352) and culicine mosquitoes (F = 0.600, df 2, P = 0.557), while there were no fed *An. gambiae *collected by the traps.

**Table 4:** Comparison of the mean catch per trap per night for each of the three abdominal status of each mosquito species collected by the three CFG traps used in comparative studies using counterflow geometry traps in Lwanda Nyamasari village.

		*Anopheles gambiae*				*Anopheles funestus*				Culicines				
**Trap**	**N**	**Fed** **mean**	**Unfed** **mean**	**Gravid** **mean**	**Sum** **%**	**Fed** **mean**	**Unfed** **mean**	**Gravid** **mean**	**Sum** **%**	**Fed** **mean**	**Unfed** **mean**	**Gravid** **mean**	**Sum** **%**	**Total No. of mosquitoes** **%**

MC	9	0.0^a^	1.4^ab^	0.0^a^	13(36)	0.2^a^	3.4^b^	0^a^	33(59)	0.3^a^	0.9^b^	0.0^a^	11(52)	57(50)

LC	9	0.0^a^	2.4^b^	0.1^a^	23(64)	0.1^a^	2.4^ab^	0.0^a^	23 (41)	0.1^a^	1.0^b^	0.0^a^	10(48)	56(50)

NB	9	0.0^a^	0.0^a^	0.0^a^	0 (0)	0.0^a^	0.0^a^	0.0^a^	0(0)	0.0^a^	0.0^a^	0.0^a^	0 (0)	0(0)

Sum of each mosquito species in each trap is also shown with the percentage in parenthesis.

**MC**, counterflow geometry trap baited with milk cream; **LC**, counterflow geometry trap baited with Limburger cheese; **NB**, counterflow geometry trap with no bait. **N **represents the number of days. The percentages are calculated for each mosquito species. For example the counterflow geometry trap baited with milk cream collected 36% of all the *An. gambiae s.l*, collected by the three traps while, the counterflow geometry trap baited with Limburger cheese collected 64% of all the same.

RETRACTED

Values following each other in the same column with different letter superscripts are significantly different at (P = 0.05).

Also, the trapping method had no significance on the trap efficacy in trapping gravid *An. gambiae*, (F = 1.000, df 2, P = 0.383), *An. funestus *and culicines as there were no gravid *An. funestus *and culicine mosquitoes collected.

The trapping method had significance on the trap efficacy in trapping unfed *An. funestus *(P = F = 3.654, df 2, P = 0.041) and unfed culicine mosquitoes (F = 5.756, df 2, P = 0.009) but not unfed *An. gambiae *(F = 3.309, df 2, P = 0.054). There was no significant difference in the number of unfed *An. funestus *collected by the milk cream baited trap and the Limburger cheese baited trap (P = 0.613). This trend was followed for the *An. gambiae *and culicine mosquitoes. However, the milk cream baited trap collected significantly higher numbers of unfed *An. funestus *than the trap with no bait (P = 0.017) while there was no significant difference in the unfed *An. funestus *collected by the Limburger cheese baited trap (P = 0.052) and the no bait trap. The Limburger cheese baited trap collected a significantly higher number of unfed *An. gambiae *than the trap with no bait (P = 0.022) while there was no significant difference between the unfed *An. gambiae *collected by the trap baited with milk cream and the trap with no bait (P = 0.069). Both the milk cream baited trap and the Limburger cheese baited trap collected significantly higher numbers of unfed culicine mosquitoes than the trap with no bait (P = 0.022) and (P = 0.003) respectively.

#### Comparative efficacy studies using CDC light traps

The mean catches of mosquitoes for each species trapped by each trapping method per night are shown in Figure 3. The trapping method had significance on the trap efficacy in trapping *An. funestus *(F = 5.169, df 3, P < 0.001), *An. gambiae *(F = 10.702, df 3, P < 0.001,) and culicine mosquitoes (F = 3.321, df 3, P = 0.021) The CDC light trap with light on collected significantly more *An. funestus *than the milk cream baited trap (P = 0.002) the Limburger cheese baited trap, (P = 0.018) and the not baited trap (P < 0.001) while there was no significant difference between the milk cream baited trap and the Limburger cheese baited trap with the trap with no bait (P = 0.663 and 0.225) respectively. There was also no significant difference in the number of *An*. *funestus *collected by the milk cream baited trap and the Limburger cheese baited trap (P = 0.436). This trend was also followed for the *An. gambiae *and culicine mosquitoes.

RETRACTED

**Figure 3:** **Comparison of different trapping methods used in the comparative studies using centers for disease control light traps**. Average number of female mosquitoes caught per trap per night. The alphabetical symbols, **a **and **b **are used to represent differences as determined by unianova test. Trapping efficiencies for the different trapping methods in collecting a certain species are not significantly different (P = 0.05), if the bars representing a particular species in each trap share any of these alphabets. The Y-error bars represent 95% confidence intervals. **LC**, CDC light trap baited with Limburger cheese; **LT**, CDC light trap baited with light on; **MC**, CDC light trap baited with milk cream; **NB**, CDC light trap NOT baited.

Day had no significance in the trapping efficacy for *An. funestus *(F = 0.502, df 15, P = 0.937), *An. gambiae *(F = 1.040, df 15, P = 0.417) and culicine mosquitoes (F = 0.292, df 15, P = 996).

The mean catches per trap per night for every abdominal status for the different mosquito species are shown in Table 5. The trapping method had no significance on trap efficacy in trapping fed *An*. *funestus *(F = 1.051, df 3, P = 0.377) and fed culicine mosquitoes (F = 2.376, df 3, P = 0.079). However, the trapping method had significance on the trap efficacy in trapping fed *An. gambiae*, (F = 5.559, df 3, P = 0.002). The trap with light on collected significantly more fed *An. gambiae *than the trap baited with milk cream (P = 0.001) the trap baited with Limburger cheese (P = 0.003) and the trap with no bait (P = 0.002). It also collected significantly more fed culicines than the trap baited with Limburger cheese (P = 0.016) and the trap with no bait (P = 0.041).

**Table 5:** Comparison of the mean catch per trap per night for each of the three abdominal status of every mosquito species collected by the four CDC light traps used in the comparative studies using centers for disease control light traps at Lwanda Nyamasari village.

Trap	N	***Anopheles gambiae s.l***.				*Anopheles funestus*				Culicines				Total no of Mosquitoes, %
		**Fed** **mean**	**Unfed** **mean**	**Gravid** **mean**	**Sum** **%**	**Fed** **mean**	**Unfed** **mean**	**Gravid** **mean**	**Sum** **%**	**Fed** **mean**	**Unfed** **mean**	**Gravid** **mean**	**Sum** **%**	

MC	16	0.2^a^	5.7^a^	0.4^a^	101 (14)	0.2^a^	3.1^a^	0^a^	53 (16)	0.1^ab^	2.9^ab^	0.1^ab^	50 (20)	204 (16)

LC	16	0.3^a^	5.3^a^	0.3^a^	454 (64)	0.1^a^	4.8^a^	0.4^ab^	144 (45)	0.0^a^	2.4^a^	0.1^ab^	138 (55)	736 (57)

NB	16	0.3^a^	3^a^	0.4^a^	94 (14)	0.1^a^	2.1^a^	0.1^a^	86 (27)	0.1^a^	1.4^a^	0.0^a^	40 (16)	220 (18)

LT	16	3.9^b^	20.5^b^	3.9^b^	59 (8)	0.6^a^	7.4^b^	1.1^b^	38 (12)	0.6^b^	7.4^b^	0.6^b^	23 (9)	120 (9)

Sum of each mosquito species in each trap is also shown with the percentage in parenthesis.

RETRACTED

**MC**, CDC light trap with no light baited with milk cream; **LC**, CDC light trap with no light baited with Limburger cheese; **NB**, CDC light trap with no light and no bait; **LT**, CDC light trap with light on. **N **represents the number of days the sampling method was set. The percentages are calculated for each mosquito species. For example the CDC light trap with no light baited with milk cream collected 14% of all the *An. gambiae s.l*, collected by all the four light traps while, the CDC light trap with no light baited with Limburger cheese collected 64% of the same. Values following each other in the same column with different letter superscripts are significantly different at (P = 0.05).

The trapping method had significance on the trap efficacy in trapping gravid *An. funestus *(F = 4.405, df 3, P = 0.007), gravid *An. gambiae *(F = 5.162, df 3, P = 0.003) but not gravid culicine mosquitoes (F = 2.041, df 3, P = 0.118). The trap with light on attracted more gravid *An. funestus *than the trap baited with milk cream (P = 0.001) and the trap with no bait (P = 0.007). The trap with light on also attracted significantly more gravid *An. gambiae *than the trap baited with milk cream, the trap baited with Limburger cheese and the trap with no bait, (P = 0.004, 0.001 and 0.02) respectively.

The trapping method had significance on the trap efficacy in trapping unfed *An. funestus*, F = 4.083, df 3, P = 0.011) unfed *An. gambiae *(F = 5.442, df 3, P = 0.002) and unfed culicine mosquitoes (F = 2.728, df 3, P = 0.052). The trap with light on collected significantly more unfed *An. funestus *than the milk cream baited trap, the Limburger cheese baited trap and the trap with no bait (P = 0.012, 0.047,0.002) respectively. This same trend was followed for *An. gambiae *mosquitoes. The trap with light on also collected significantly more unfed culicines than the Limburger cheese baited trap (P = 0.049) and the trap with no bait (P = 0.008).

## Discussion

To my knowledge this is the first time that traps baited with Limburger cheese which was observed to be attractive to *An. gambiae s.s *mosquitoes in a wind tunnel bioassay [16] has successfully trapped *An. gambiae s.s*, *An. arabiensis, An. funestus *and culicine mosquitoes in the field.

RETRACTED

The current observation made on Limburger cheese contrasts with those of Murphy *et al. *[26] who found that CDC light traps baited with a synthetic mixture of Limburger cheese compounds did not catch any mosquitoes in the field. This difference in observations could be due to the fact that in their study, Murphy *et al. *[26] combined the various chemical components of Limburger cheese to bait light traps while in our work we used whole natural Limburger cheese to bait CFG traps.

This is also the first time to my knowledge that traps baited with African traditional milk cream which is also a milk product has trapped *An. gambiae s.l*, *An. funestus *and culicine mosquitoes. Considering that Knols *et al. *[27] suggested that bacteria involved in the ripening of Limburger cheese may have originated from human skin and hence that these bacteria are responsible for the production of 'human-specific' volatile organic compounds (VOCs) that mediate the host-seeking process of malaria mosquitoes as washing the feet with a bactericidal soap significantly altered the selection of biting sites of *An. gambiae *on a motionless naked volunteer [3]. It would only be sensible to suggest that one of the reasons why the milk cream was able to attract the mosquitoes was probably due to its handling by humans as skin microbes [28] which have been observed to be responsible for the odours produced by the human hosts, could have been transferred into the milk which had been used to make the milk cream.

It was also observed that CFG and CDC light traps baited with milk cream worked just as well as the same traps baited with Limburger cheese in trapping mosquitoes. This observation suggests that milk cream could be used in place of Limburger cheese and *vice versa *though more studies should be done for reproducible results.

There was no significant difference in the numbers of *An. funestus *caught by the CFG trap baited with Limburger cheese from the numbers caught by man-landing catches (MLC). This observation suggests that Limburger cheese baited traps would provide an efficient alternative to MLC during surveillance and monitoring of malaria vectors during epidemiological studies. It was also observed that the CFG trap baited with Limburger cheese collected higher proportions of parous *An. arabiensis*, *An. gambiae *and *An. funestus *than the CDC light trap, the entry trap and the MLC. This observation suggests that the CFG trap collects higher proportions of parasite infected mosquitoes as earlier studies have shown that parous mosquitoes have higher sporozoite infections than the nulliparous ones [29].

RETRACTED

Furthermore, the Limburger cheese baited CFG trap collected larger *An. gambiae *than the CDC trap, the entry trap and the MLC. This observation could also suggests that the Limburger cheese baited trap collected *An. gambiae *mosquitoes that have a higher vector competence and vectorial capacity, as studies before have suggested that larger mosquitoes tend to have more serial feeding than small ones and are therefore likely to infect more hosts than the small ones[30]. Earlier studies also observed that larger mosquitoes have a higher probability of survival, being inseminated and producing more egg batches than smaller ones [31].

It was also observed that the Limburger cheese-baited CFG trap was biased in catching gravid *An. funestus *when compared with man-landing catches. This indicates that the Limburger cheese would provide a good odour bait in oviposition traps especially for *An. funestus *as it has been observed that mosquitoes locate their oviposition sites via chemical attractants [32].

The Limburger cheese-baited CFG trap, like the man-landing catches and the CDC light trap attracted higher numbers of *An. gambiae*, *An. arabiensis *and *An. funestus *than the entry trap. This could be explained by the fact that while the entry trap is fixed at an open window some host-seeking mosquitoes could be entering the house through the door and the eaves which are the most important entry points for mosquitoes that spread malaria and a variety of tropical diseases. Some could also be entering into the house earlier before the entry trap is placed onto a window. The entry trap therefore, is not an effective method for sampling Afrotropical malaria vectors according to this study.

## Conclusions

In this study, Limburger cheese and milk cream have demonstrated a potential as odour baits that can be used as an alternative to the unethical man-landing catches in sampling and monitoring the African malaria vector *An. funestus *in the field. Limburger cheese has also shown a potential as an effective odour bait in trapping gravid *An. funestus *and one could even foresee the use of Limburger cheese as an attractant in oviposition traps for *An. funestus *mosquitoes. However, it might be prudent to combine odours from Limburger cheese or milk cream with other chemical cues which also play a role in host identification and location mainly components of the human sweat - ammonia, lactic acid and carboxylic acids - [33,34] and breath [2] in order to develop a highly attractive odour blend that can be used in the control of mosquitoes. It would also be important to set up the experiments from 18.00 h to 06.00 h to accommodate the two blood seeking cycles (sunset and sunrise) in mosquitoes [23] unlike in this study where the traps were set at 22.00 h to 06.00 h and therefore only one cycle was covered.

RETRACTED

## Competing interests

The authors declare that they have no competing interests.

## Authors' contributions

EAO conceived, designed, performed the experiments and analyzed the data.
